The article "Correlation Analysis between the Viral Load and the Progression of COVID-19" was published in 2021. Journal: Comput Math Methods Med.

# Correlation Analysis between the Viral Load and the Progression of COVID-19

**DOI:** 10.1155/2021/9926249

**Published:** 2021-06-08

**Authors:** Wenyu Chen, Qinfeng Xiao, Zhixian Fang, Xiaodong Lv, Ming Yao, Min Deng

**Affiliations:** ^1^Department of Respiration, Affiliated Hospital of Jiaxing University/The First Hospital of Jiaxing, Jiaxing 314000, China; ^2^Center for Pain Medicine, Affiliated Hospital of Jiaxing University/The First Hospital of Jiaxing, Jiaxing 314000, China; ^3^Department of Infectious Disease, Affiliated Hospital of Jiaxing University/The First Hospital of Jiaxing, Jiaxing 314000, China

## Abstract

**Objectives:**

This study is aimed at exploring the relationship of the viral load of coronavirus disease 2019 (COVID-19) with lymphocyte count, neutrophil count, and C-reactive protein (CRP) and investigating the dynamic change of patients' viral load during the conversion from mild COVID-19 to severe COVID-19, so as to clarify the correlation between the viral load and progression of COVID-19.

**Methods:**

This paper included 38 COVID-19 patients admitted to the First Hospital of Jiaxing from January 28, 2020, to March 6, 2020, and they were clinically classified according to the Guidelines on the Novel Coronavirus-Infected Pneumonia Diagnosis and Treatment. According to the instructions of the Nucleic Acid Detection Kit for the 2019 novel coronavirus (SARS-CoV-2), respiratory tract specimens (throat swabs) were collected from patients for nucleic acid testing. Patients' lymphocyte count and neutrophil count were determined by blood routine examination, and CRP was measured by biochemical test.

**Results:**

The results of our study suggested that the cycle threshold (Ct) value of Nucleocapsid protein (N) gene examined by nucleic acid test was markedly positively correlated with lymphocyte count (*p* = 0.0445, *R*^2^ = 0.1203), but negatively correlated with neutrophil count (*p* = 0.0446, *R*^2^ = 0.1167) and CRP (*p* = 0.0393, *R*^2^ = 0.1261), which indicated that patients with a higher viral load tended to have lower lymphocyte count but higher neutrophil count and CRP. Additionally, we detected the dynamic change of Ct value in patients who developed into a severe case, finding that viral load of 3 patients increased before disease progression, whereas this phenomenon was not found in 2 patients with underlying diseases.

**Conclusion:**

The results of this study demonstrated that viral load of SARS-CoV-2 is significantly negatively correlated with lymphocyte count, but markedly positively correlated with neutrophil count and CRP. The rise of viral load is very likely to be the key factor leading to the overloading of the body's immune response and resulting in the disease progression into severe disease.

The article "Correlation Analysis between the Viral Load and the Progression of COVID-19" was published in 2021. Journal: Comput Math Methods Med.

## 1. Introduction

Since the outbreak of novel coronavirus pneumonia in Wuhan, Hubei Province, China, in December 2019 [1–3], the epidemic swept the whole country and other nations in the world and has been lasting till now [4–6]. At the early stage of the epidemic, China's public health system and clinical and scientific circles acted quickly in order to timely identify the novel virus and publicize the gene sequence of the virus to the world [7]. On February 12, 2020, the disease was officially named coronavirus disease 2019 (COVID-19) by World Health Organization (WHO). The most common symptoms of COVID-19 are fever, cough, myalgia, fatigue, pneumonia, and dyspnea, while a few patients have headache, diarrhea, hemoptysis, runny nose, expectoration, etc. [8, 9]. Besides, the diagnosis of asymptomatic COVID-19 patients is also a tough issue. For suspected cases, they are generally confirmed upon positive nucleic acid testing for the 2019 novel coronavirus (SARS-CoV-2) in sputum, throat swab, and lower respiration secretion by means of real-time fluorescence PCR (RT-PCR). RT-PCR can efficiently and quickly finish detecting virus samples, with high sensitivity and specificity. Hence, it has become the first detection method recommended in the Guidelines on the Novel Coronavirus-Infected Pneumonia Diagnosis and Treatment (6^th^ edition) [10].

SARS-CoV-2 is a positive-stranded RNA (+RNA) virus and belongs to *Coronaviridae* family, *Nidovirales* order. Coronaviruses can infect the respiratory system, gastrointestinal tract, liver, and central nervous system of humans, mammals, birds, bats, etc. [11, 12]. The positive single-stranded RNA genome of the SARS-CoV-2 is about 30 k nucleotides in size, encoding 9,860 amino acids [7, 13, 14]. Traditionally, the preferred targets for RT-PCR detection of coronavirus include conversed or largely expressed genes such as structural Spike glycoprotein (S) and Nucleocapsid protein (N) genes and unstructural RdRp and replicase open reading frame (ORF) 1ab genes [12]. Fluorescence RT-PCR can be performed to detect the cycle threshold (Ct) values of these genes, which could be used to represent viral load, as there is a negative correlation between Ct value and virus RNA copy number [15].

Recently, some researchers have reported the correlation between the viral load and disease progression and spread. A retrospective study by Xu et al. [16] suggested that Ct values detected from the tertiary patients at the time of admission were similar to those from the Wuhan imported and secondary cases (both *p* > 0.05). For the tertiary group, the viral load was undetectable for all patients on day 14. For 1/3 of the patients in the imported and secondary groups, the viral load remained positive on day 14 after the admission, which indicated that the tertiary patients were gradually less susceptible to SARS-CoV-2 infection. Another research unveiled that the viral load of COVID-19 patients' sputum peaked in the 1^st^ week after the appearance of symptoms, but that decreased with time going by. Besides, the older people tended to have a higher viral load. Different from the severe acute respiratory syndrome (SARS), patients with COVID-19 have a higher viral load, which may account for the fast spread of the epidemic [17]. The infection mode of SARS-CoV-2 is completely different from SARS. For SARS, the incubation period is not contagious. Generally, the virus RNA level in vivo reaches its peak 7-10 d after the onset of symptoms, while for SARS-CoV-2, the RNA level reaches its peak within 5 d of the onset of symptoms and replicates actively in the upper respiratory tract tissue, indicating that people infected with COVID-19 shed or spread the virus in large quantities within the first 5 d of the onset of symptoms [18]. Therefore, infected patients with mild symptoms or even asymptomatic stages are particularly important for epidemic prevention and control. Currently, the relationship between the viral load and severity of disease of COVID-19 patients has not been fully understood. Although there is research suggesting that COVID-19 patients with severe disease conditions need to be treated in intensive care unit (ICU), and they have a relatively higher viral load [15], yet the time of exacerbation for these patients in the pathogenic process remains unclear. As a result, it is crucial to continue exploring the correlation between the viral load and development of COVID-19, which helps to better monitor disease progression and is of certain guiding significance for the treatment and prevention of COVID-19.

The article "Correlation Analysis between the Viral Load and the Progression of COVID-19" was published in 2021. Journal: Comput Math Methods Med.

In this study, we detected the Ct values of N gene and ORF 1ab gene of 38 patients through the SARS-CoV-2 Nucleic Acid Detection Kit (Sansure Biotech Inc., China) and analyzed the correlation between these Ct values and lymphocyte count, neutrophil count, and C-reactive protein (CRP). Meanwhile, we applied a dynamic detection towards the Ct value of N gene in mild patients who developed into a severe case later aiming to evaluate the change of Ct value during the disease progression, so as to provide evidence for the correlation between the viral load and disease progression.

## 2. Materials and Methods

### 2.1. Information Collection

This paper included 38 COVID-19 patients admitted to the First Hospital of Jiaxing and The First Affiliated Hospital, Zhejiang University School of Medicine from January 28, 2020, to March 6, 2020, with the highest temperature reaching 37-39.6°C. Nucleic acid samples were collected from the patients' respiratory tracts and detected by qRT-PCR, indicating RNA positive. The patients included 22 males and 16 females, with the average age being 47.37 ± 13.27 years old.

According to the Guidelines on the Novel Coronavirus-Infected Pneumonia Diagnosis and Treatment (7^th^ edition) [19], we classified the patients into the following: (1) mild group: having mild clinical symptoms, with no sign of pneumonia observed in imaging; (2) moderate group: having fever and respiratory symptoms, with signs of pneumonia observed in imaging; (3) severe group: adults who have any one of the following symptoms are classified into the severe group: having dyspnea, respiratory rate (RR) ≥ 30 breaths/min or oxygen saturation (SpO2) ≤ 93% at resting state or arterial partial pressure of oxygen (PaO2)/oxygen concentration (FiO2) ≤ 300 mmHg; pulmonary imaging shows marked lesion progression > 50% within 24-48 h; (4) critically severe group: patients who have any one of the following symptoms need to be sent to ICU: having respiratory failure and needing mechanical ventilation or having shock or combined with other organ failures. Here, patients of mild and moderate types were named mild patients, and patients of severe and critically severe types were named severe patients. There was 1 severe case and 37 mild cases at the time of admission, and 7 mild cases developed into a severe case later.

### 2.2. Sample Collection and Preservation

The respiratory samples (throat swabs) and blood samples of the subjects were collected by the First Hospital of Jiaxing according to the technical guidance for laboratory testing of COVID-19. Respiratory samples were preserved at 4°C and detected within 24 h. Blood samples were preserved at -20°C. All samples were preserved in a specially made refrigerator, taken care of by people who were specially assigned, and destroyed when the experiment ended.

### 2.3. Nucleic Acid Extraction and Detection

RNA from the respiratory samples was gradually extracted using the SARS-CoV-2 Nucleic Acid Detection Kit (Sansure Biotech Inc., China). qRT-PCR was employed to detect the ORF 1ab and N genes, with the operation methods and result interpretation following the manufacturer's instructions. The suspicious results were notified to the clinic for resampling and reexamination. One of the target genes in the same sample being positive meant the sample was SARS-CoV-2 positive, but negative if both two genes were negative. In this study, we used the Ct value of N gene as a reference. The Ct value was inversely correlated with RNA copy number of virus [15]. Ct value < 40 was considered COVID-19 positive.

The article "Correlation Analysis between the Viral Load and the Progression of COVID-19" was published in 2021. Journal: Comput Math Methods Med.

### 2.4. Other Detection Indexes

1. *Blood Routine Indexes*. The changes of patients' blood routine indexes were detected every 2-7 d, especially the neutrophil (10^9^/L) and lymphocyte count (10^9^/L).
2. *Biochemical Indexes*. The changes of patients' biochemical indexes were detected every 2-7 d, especially CRP (mg/L).

### 2.5. Statistical Analysis

All the data were processed using the Graphpad Prism 8.0 software. Linear regression analysis was used as correlation analysis, and *p* values and *R*^2^ values were calculated. Part of the enumeration data was expressed as mean ± standard deviation (SD) and analyzed by Student's *t*-test. *p* < 0.05 was considered statistically significant.

## 3. Results

### 3.1. Correlation between the Ct Value of Viral RNA and Neutrophil, Lymphocyte Count, and CRP in COVID-19 Patients

Pneumonia virus infection tends to cause the abnormality of CRP and some blood routine indexes. In order to investigate the relationship of the Ct value of viral RNA with neutrophil, lymphocyte count, and CRP in COVID-19 patients, we performed a linear regression analysis. Firstly, we eliminated the samples (*n* = 4; 3; 4) whose nucleic acid detection time did not match their blood test time and analyzed the data of the rest of the samples (*n* = 34; 35; 34). As can be seen from the results, the Ct value determined by nucleic acid detection was markedly positively correlated with lymphocyte count (Figure 1(a), *p* < 0.05) but significantly negatively correlated with neutrophil count and CRP (Figures 1(b) and 1(c), *p* < 0.05). The lower Ct values generally represent the higher viral load. Consequently, we speculated that patients with a higher viral load tended to have increased CRP and neutrophil count but decreased lymphocyte count. Hypersensitive CRP (hs-CRP) is a nonspecific marker in the acute phase of systemic inflammatory response [20, 21]. Body injury induced by increased viral load triggers the sharp rise in CRP level, and CRP elevation could promote the motion of neutrophil and macrophages, inhibit mixed lymphocyte reaction, and induce inflammatory response in body to resist virus invasion. In addition, various researches have revealed that the number of lymphocytes is negatively correlated with degree of inflammation [22, 23]. Therefore, increased CRP and decreased lymphocyte both indicated worsening of inflammation, demonstrating that increased viral load would be accompanied by excessive inflammation, which is highly likely to be the key factor contributing to the induction of cytokine storm and development of disease.

The article "Correlation Analysis between the Viral Load and the Progression of COVID-19" was published in 2021. Journal: Comput Math Methods Med.

### 3.2. The Change in Nucleic Acid Ct Value of Severe COVID-19 Patients

In order to further explore the change of Ct value during the disease progression, mild patients who developed into a severe case and did nucleic acid detection at least 4 times were included and 5 samples were obtained. These patients' symptoms gradually became severe, and patients developed into a severe case 5-10 d after being confirmed (Figures 2(a)–2(e)). It could be seen from the results that most patients' Ct values had a decreasing tendency before or during the severe conversion, and the values were generally low, which revealed that they had a higher viral load. In the meantime, their symptoms gradually deteriorated with the continual rise in viral load (Figures 2(b), 2(c) and 2(e)). However, other 2 patients had a higher Ct value when converting to severe cases. That is to say, their viral load was not high and did not rise when patients developed into a severe case, but they were found to be aged people and had underlying diseases. One patient had diabetes (Figure 2(a)), and another one had hyperlipidemia (Figure 2(d)) and had a trend to recur. Therefore, their poor physical quality was highly likely to be the key factor driving their disease progression. The above results indicated that most severe patients' viral load tended to increase with the deterioration of the disease, whereas the immunity and physical quality of some patients also affected the disease progression. Accordingly, although the viral load is able to partially predict patients' disease progression, it is not the only basis.

## 4. Conclusion

This study firstly investigated the correlation between the viral load and part of the blood routine indexes (neutrophil and lymphocyte count) and CRP in COVID-19 patients. These 3 indexes could predict the occurrence of body inflammation. Many researchers suggested that early COVID-19 cases generally have normal or decreased leukocyte and reduced lymphocyte, and most patients have increased hs-CRP and normal PCT. For example, Zhou et al. conducted a retrospective study based on 62 laboratory-confirmed cases, finding that 24 out of 30 patients (80%) had a decreased lymphocyte count after blood routine examination; 18 out of 27 cases (66.7%) had an increased erythrocyte sedimentation rate (ESR), and 27 cases (100%) had increased hs-CRP regarding ESR and hs-CRP detection [24]. Similar results were observed in another retrospective analysis concerning COVID-19 patients: most patients had a reduced lymphocyte count (33/51, 65%), while a few patients had a normal one (17/51, 35%) [25]. Besides, research unveiled that among the 452 included COVID-19 patients, 286 were diagnosed as seriously infected and they tended to have a lower lymphocyte count [26]. In our research, we performed a retrospective analysis aiming to explore the correlation between the lymphocyte count and Ct value of 38 COVID-19 patients, the result of which uncovered that they were markedly positively correlated, meaning that patients' lymphocyte count had a falling tendency with the rise of the viral load in respiratory tracts. This may partially explain the reason why most COVID-19 patients had a reduced lymphocyte count.

The article "Correlation Analysis between the Viral Load and the Progression of COVID-19" was published in 2021. Journal: Comput Math Methods Med.

CRP is a type of sharply risen protein (acute protein) in plasma when body is infected or tissue is injured, which leads to opsonization by activating complement and promoting the phagocytosis of phagocyte and is able to clear away the pathogenic microorganism that invades body. Research has found that CRP level is positively correlated with the diameter of lung lesions and could reflect disease severity of COVID-19 patients [27]. In addition, Liu et al. [28] discovered that the increase of neutrophil, SAA, PCT, CRP, cTnI, D-dimer, LDH, and lactate levels could indicate COVID-19 progression and decreased lymphocyte count. These researches have revealed that increased CRP level is associated with disease progression. Besides, we found that a higher viral load (lower Ct value) corresponded with a higher CRP level.

Neutrophils are one of the important immune cells which can be quickly accumulated to sites of infection to play their role in host defense and immunoregulation [29]. Some retrospective studies have explored the relationship between body internal change of neutrophils and COVID-19. For instance, research unveiled that patients who had ocular symptoms were more likely to have higher leukocyte and neutrophil count compared with those who had no ocular symptoms [30]. Besides, research has explored the potential biomarkers which are capable of predicting disease severity by analyzing the epidemiological, clinical, laboratory, and radiological features of COVID-19 patients in Shenzhen, China, among which viral load and neutrophil ratio are both likely to be the predictors of disease severity [28]. In the present study, we found that Ct value might have a negative linear correlation with neutrophil count, which meant that viral load might have a positive linear correlation with neutrophil count. This suggested that higher viral load corresponded with higher neutrophil count.

The sudden deterioration, shock, and hypoxemia of COVID-19 may be related to cytokine storm [31]. Huang et al. [32] discovered that patients who entered ICU had a higher level of IL2, IL7, IL10, GSCF, IP10, MCP1, MIP1A, TNF*α*, and other inflammatory factors in plasma than those who were in routine ward, which reflected from one aspect that severe and critically severe patients had marked inflammatory response. Consequently, apart from exploring the correlation between viral load and inflammatory indexes, this paper further detected the dynamic change in Ct value of mild patients who developed into a severe case so as to clarify the viral load change before and after severe conversion. Research published in New England Journal of Medicine indicated that SARS-CoV-2 mainly spreads 2 d after the onset of the disease, and viral load in respiratory tracts is moderate in the early period but peaks about 10 d after the onset of the disease [15]. A study demonstrated that viral load is likely to become one of the predictors for disease progression [28]. Among the 7 mild cases included in our hospital who developed into a severe case later, 5 patients had complete data of nucleic acid detection, and these 5 patients developed into a severe case within 5-10 d after being confirmed. Among these 5 cases, 3 patients' Ct values showed a falling tendency, which suggested that their viral load gradually increased. Although the other 2 cases accompanied by underlying diseases had a decreased viral load in early period of treatment, they developed into a severe case after a time, and their viral load rose again after the conversion. These results indicated that despite the correlation between increased viral load and disease exacerbation, the former was not necessarily the only factor contributing to the latter.

The article "Correlation Analysis between the Viral Load and the Progression of COVID-19" was published in 2021. Journal: Comput Math Methods Med.

Taken together, through analysis on part of the blood routine indexes, biochemical indexes, and nucleic acid Ct values of COVID-19 patients treated in our hospital, our retrospective study found that patients' viral load of SARS-CoV-2 was negatively correlated with lymphocyte count but positively correlated with neutrophil count and CRP. These indexes may be associated with patients' inflammation and are likely to be employed to predict disease progression. Additionally, we discovered that some patients' viral load tended to increase during the conversion from mild cases to severe cases, but it was not the only reason for the deterioration of the disease. As every coin has two sides, there are some limitations in the present study. For example, this study is a single-center retrospective study, with a small sample size. Some sample data are incomplete, and patients cannot be dynamically monitored throughout the course of the disease. Due to the small number of cases and the low *R*^2^ values in correlational results, the results might deviate from the experiments. Besides, we were also short of severe cases, and the data of some patients' whole course of disease could not be accessed. Hence, a large sample, multicenter study is warranted.

The article "Correlation Analysis between the Viral Load and the Progression of COVID-19" was published in 2021. Journal: Comput Math Methods Med.

## Figures and Tables

**Figure 1:** Correlation between the Ct value of viral RNA and lymphocyte count, neutrophil count, and CRP in COVID-19 patients. Correlation analysis on the Ct value of viral RNA and (a) lymphocyte count (*R*^2^ = 0.1203, *p* = 0.0445, and *n* = 34), (b) CRP (*R*^2^ = 0.1167, *p* = 0.0446, and *n* = 35), and (c) neutrophil count (*R*^2^ = 0.1261, *p* = 0.0393, and *n* = 34) in COVID-19 patients.

**Figure 2:** The change of nucleic acid Ct value in severe COVID-19 patients. (a–e) 5 patients' Ct value changes with time going by during the treatment. Red line refers to the time and Ct value when mild COVID-19 patients developed into a severe case.

## Data Availability

The data and materials in the current study are available from the corresponding author on reasonable request.

## References

[1] Zu Z. Y., Di Jiang M., Xu P. P. (2020). Coronavirus disease 2019 (COVID-19): a perspective from China. *Radiology*.

[2] Chen H., Guo J., Wang C. (2020). Clinical characteristics and intrauterine vertical transmission potential of COVID-19 infection in nine pregnant women: a retrospective review of medical records. *The Lancet*.

[3] Shi H., Han X., Jiang N. (2020). Radiological findings from 81 patients with COVID-19 pneumonia in Wuhan, China: a descriptive study. *The Lancet Infectious Diseases*.

[4] Yi Y., Lagniton P. N. P., Ye S., Li E., Xu R. H. (2020). COVID-19: what has been learned and to be learned about the novel coronavirus disease. *International Journal of Biological Sciences*.

[5] CDC COVID-19 Response Team, Bialek S., Boundy E. (2020). Severe outcomes among patients with coronavirus disease 2019 (COVID-19) - United States, February 12–March 16, 2020. *MMWR. Morbidity and Mortality Weekly Report*.

[6] Spiteri G., Fielding J., Diercke M. (2020). First cases of coronavirus disease 2019 (COVID-19) in the WHO European Region, 24 January to 21 February 2020. *Euro Surveillance*.

[7] Chan J. F.-W., Yuan S., Kok K.-H. (2020). A familial cluster of pneumonia associated with the 2019 novel coronavirus indicating person-to-person transmission: a study of a family cluster. *The Lancet*.

[8] Rothan H. A., Byrareddy S. N. (2020). The epidemiology and pathogenesis of coronavirus disease (COVID-19) outbreak. *Journal of Autoimmunity*.

[9] Lai C. C., Shih T. P., Ko W. C., Tang H. J., Hsueh P. R. (2020). Severe acute respiratory syndrome coronavirus 2 (SARS-CoV-2) and coronavirus disease-2019 (COVID-19): the epidemic and the challenges. *International Journal of Antimicrobial Agents*.

The article "Correlation Analysis between the Viral Load and the Progression of COVID-19" was published in 2021. Journal: Comput Math Methods Med.

[10] General Office of National Health Commission of the People’s Republic of China (2020). *Guidelines on the Novel Coronavirus-Infected Pneumonia Diagnosis and Treatment*.

[11] de Wilde A. H., Snijder E. J., Kikkert M., van Hemert M. J. (2017). Host factors in coronavirus replication. *Current Topics in Microbiology and Immunology*.

[12] Cui J., Li F., Shi Z. L. (2019). Origin and evolution of pathogenic coronaviruses. *Nature Reviews. Microbiology*.

[13] Chan J. F.-W., Kok K.-H., Zhu Z. (2020). Genomic characterization of the 2019 novel human-pathogenic coronavirus isolated from a patient with atypical pneumonia after visiting Wuhan. *Emerging Microbes & Infections*.

[14] Lu R., Zhao X., Li J. (2020). Genomic characterisation and epidemiology of 2019 novel coronavirus: implications for virus origins and receptor binding. *The Lancet*.

[15] Zou L., Ruan F., Huang M. (2020). SARS-CoV-2 viral load in upper respiratory specimens of infected patients. *The New England Journal of Medicine*.

[16] Xu T., Chen C., Zhu Z. (2020). Clinical features and dynamics of viral load in imported and non-imported patients with COVID-19. *International Journal of Infectious Diseases*.

[17] To K. K.-W., Tsang O. T.-Y., Leung W.-S. (2020). Temporal profiles of viral load in posterior oropharyngeal saliva samples and serum antibody responses during infection by SARS-CoV-2: an observational cohort study. *The Lancet Infectious Diseases*.

[18] Wölfel R., Corman V. M., Guggemos W. (2020). Virological assessment of hospitalized patients with COVID-2019. *Nature*.

[19] General Office of National Health Commission of the People’s Republic of China (2020). *Guidelines on the Novel Coronavirus-Infected Pneumonia Diagnosis and Treatment*.

[20] Iglesias-Álvarez D., López-Otero D., González-Ferreiro R. (2018). Prognostic value of hs-CRP after transcatheter aortic valve implantation. *Circulation: Cardiovascular Interventions*.

[21] Ding G. Z., Li W. S. (2018). The expressions and significance of APN, D-D, IL-17 and hs-CRP in patients with acute exacerbation of chronic obstructive pulmonary disease. *European Review for Medical and Pharmacological Sciences*.

[22] Prats-Puig A., Gispert-Saüch M., Díaz-Roldán F. (2015). Neutrophil-to-lymphocyte ratio: an inflammation marker related to cardiovascular risk in children. *Thrombosis and Haemostasis*.

[23] Yilmaz G., Sevinc C., Ustundag S. (2017). The relationship between mean platelet volume and neutrophil/lymphocyte ratio with inflammation and proteinuria in chronic kidney disease. *Saudi Journal of Kidney Diseases and Transplantation*.

[24] Zhou S., Wang Y., Zhu T., Xia L. (2020). CT features of coronavirus disease 2019 (COVID-19) pneumonia in 62 patients in Wuhan, China. *American Journal of Roentgenology*.

The article "Correlation Analysis between the Viral Load and the Progression of COVID-19" was published in 2021. Journal: Comput Math Methods Med.

[25] Song F., Shi N., Shan F. (2020). Emerging 2019 novel coronavirus (2019-nCoV) pneumonia. *Radiology*.

[26] Qin C., Zhou L., Hu Z. (2020). Dysregulation of immune response in patients with COVID-19 in Wuhan, China. *Clinical Infectious Diseases*.

[27] Wang L. (2020). C-reactive protein levels in the early stage of COVID-19. *Médecine et Maladies Infectieuses*.

[28] Liu Y., Yang Y., Zhang C. (2020). Clinical and biochemical indexes from 2019-nCoV infected patients linked to viral loads and lung injury. *Science China. Life Sciences*.

[29] Liew P. X., Kubes P. (2019). The neutrophil's role during health and disease. *Physiological Reviews*.

[30] Wu P., Duan F., Luo C. (2020). Characteristics of ocular findings of patients with coronavirus disease 2019 (COVID-19) in Hubei Province, China. *JAMA Ophthalmology*.

[31] Xu K., Cai H., Shen Y. (2020). Management of corona virus disease-19 (COVID-19): the Zhejiang experience. *Zhejiang Da Xue Xue Bao Yi Xue Ban*.

[32] Huang C., Wang Y., Li X. (2020). Clinical features of patients infected with 2019 novel coronavirus in Wuhan, China. *The Lancet*.

